The article "Application of Clinical Case Teaching Mode in Gynecological Nursing Teaching" was retracted in 2023. Reasons: unreliable results or conclusions; lack of ethics approval or compliance; concerns about the data; concerns about the peer review.

# Application of Clinical Case Teaching Mode in Gynecological Nursing Teaching

**DOI:** 10.1155/2022/9739313

**Published:** 2022-08-10

**Authors:** Yining Mei

**Affiliations:** School of Nursing, Ningbo College of Health Sciences, Ningbo 315100, China

## Abstract

**Background:**

Looking at the existing literature, it can be found that the clinical case teaching method is widely used in most majors, but it is rarely used in the field of gynecological nursing teaching. Seriously restrict the progress of gynecological nursing teaching in practice.

**Objective:**

To explore the application and effect of clinical case teaching mode in gynecological nursing teaching.

**Methods:**

Two classes of gynecological nursing courses in midwifery majors in 2019 were selected as the research objects. The experimental group was taught by the clinical case teaching mode, while the control group was taught by the traditional teaching mode.

**Results:**

The students in the experimental group were better than those in the control group, with a statistically significant difference (*P* < 0.05); the students in the experimental group were better than the control group in the evaluation of classroom effects, and the difference was statistically significant (*P* < 0.05).

**Conclusion:**

The application of clinical case teaching mode in gynecological nursing teaching is beneficial to the improvement of students' performance, to stimulate students' interest in learning, and to improve their self-learning ability, clinical thinking, analysis and problem solving, teamwork, and communication skills. The clinical case teaching mode has played an active role in gynecological nursing teaching, which is well received by students and is worthy of promotion.

## 1. Introduction

Clinical case teaching guides students to obtain the expected effect of classroom teaching through active thinking and exploration by taking specific real cases as the analysis object [1–9]. In this mode, students can have a more scientific understanding of the subject of the classroom and will also have a clear impression of the specific application of theoretical knowledge. Because of its advantages in improving students' operational skills and practical level, clinical case teaching has been widely adopted in recent years [10, 11]. This change has, to a large extent, reversed the learning model in which teachers occupy the core of the classroom and students passively listen to lectures and memorize knowledge points in our country's education. Through the thinking and arrangement of each link in the case, the students verified the existing theoretical knowledge and enhanced their enthusiasm for professional learning. Gynecological nursing is an important professional ability quality course for nursing majors, and it is also a clinical nursing course that closely combines theory and practice [12, 13]. With good communication skills, careful clinical thinking skills, keen observation skills, and strong adaptability, it will lay a good foundation for future clinical nursing work and career development. However, compared with other courses, the characteristics of gynecological nursing pose challenges to teaching [14, 15]. For example, the object of gynecological nursing is the female reproductive system, which involves privacy and puts forward higher requirements on the communication ability of nurses and patients. In addition, there are many emergencies such as ectopic pregnancy, ovarian cyst pedicle torsion, rupture, etc.; clinical cases such as endocrine diseases and tumor diseases are complex and changeable. These are the difficulties encountered by students in the learning process [16, 17]. At this stage, based on the Internet of Things technology, students can simulate and observe the surgical process in all directions from many perspectives, so that they have a more scientific understanding of the main points and difficulties of the surgical process. How to improve the quality and effect of gynecological nursing teaching is a hot issue that scholars pay attention to [18].

In this study, the clinical case teaching model was introduced into the gynecological nursing teaching process. The main method adopted in the research is the comparative research method. For example, in the teaching of nursing after uterine fibroids, the evaluation of traditional teaching will only be based on the nursing points. In the case teaching mode, with the help of the virtual scene constructed by the Internet of Things, various postoperative situations can be carried out. Simulation was done, so as to realize the investigation of students' overall ability. The following steps were generally taken: after determining the teaching objectives, teachers optimized the real situation before class to form a model suitable for students, which could guide students to think and make decisions [19]. The case is used as a classroom explanation material or practice thinking to arrange for students and guide them to understand the case through independent research, group discussion, etc., and strengthen the grasp of the link. The purpose of this teaching mode is to free students from boring theoretical lectures, to be close to clinical practice, to focus on cultivating students' clinical thinking and judgment ability, ability to analyze and solve problems, to achieve seamless connection with clinical practice, and to cultivate students' job competence [20, 21]. Through experimental comparison, it is found that the clinical case teaching mode has a significant improvement in the comprehensive teaching effect compared with the traditional teaching method [22, 23]. The application process and effect are summarized as follows.

## 2. Objects and Methods

### 2.1. Research Objects

The main method adopted in the research is the comparative research method, through the comparison of the academic performance and clinical operation of the two groups of students, to explore the clinical case teaching method. Two classes of 2019 midwifery majors offering gynecological nursing courses were selected as the experimental group (46 people) and the control group (47 people), all girls, aged between 19 and 22. The two groups of learners are taught by the same teacher. The experimental group was taught by the clinical case teaching mode; the control group was taught by the traditional teaching mode [24, 25]. There was no significant difference in basic data such as gender, age, and basic course scores between the two groups (*P* > 0.05). The experimental data show that the comprehensive teaching effect of the clinical case teaching method can be improved by more than 10% compared with the traditional method. This proves that the simulation scene constructed by the Internet of Things technology through the clinical case teaching method is of great value to the improvement of teaching effect.

### 2.2. Teaching Methods

#### 2.2.1. The Experimental Group Adopts the Clinical Case Teaching Mode

The experimental group adopts the clinical case teaching mode, can be seen in Figure 1.

In Figure 2, it can be seen that at the current stage, teachers' teaching behavior can be refined into five interconnected links. Through these five links, teachers' teaching behavior improves the integrity and has a more positive impact.

- Preparation before class

Divided into several steps: (1) design and compile clinical cases. Based on the students' job competency requirements and teaching goals, teachers will select typical clinical cases, design and compile clinical cases, and form a comprehensive task learning list based on the actual work tasks. Gynecological nursing focuses on clinical practice and requires students to have certain adaptability, interpersonal communication skills, and clinical thinking and judgment skills.

Therefore, it is very important to select suitable case materials. It should be ensured that the case tasks range from simple to complex, from small tasks to large tasks, and progress through the level of clinical case tasks, so that students can evaluate the nursing of gynecological patients and raise existing nursing problems and formulate nursing plans, implement nursing measures and health education, and give nursing evaluations [26]. Finally, under the guidance of clinical cases, the purpose of knowledge connection and integration is achieved. (2) The teacher publishes the course preview package on the course online teaching platform, including learning objectives (quality objectives, knowledge objectives, and ability objectives), clinical cases (comprehensive task learning sheets), microvideos, PPT, preclass tests, and other learning resources [27]. (3) Students claim learning tasks, establish contact with their peers, and carry out corresponding learning activities for the materials, carry out in group cooperation, conduct systematic discussions around the task theme, clarify the ideas, methods and task division of solving problems, and record their own difficulties, teachers answer questions in a timely manner and check the completion of students' tasks, play a supervising role. In this process, students' autonomous learning behavior goals are reflected in stimulating intrinsic motivation, clarifying learning goals, and developing learning plans [28–30].

(b) Classroom implementation

Students are the main body and teachers are the leading concept in the classroom. (1) Student learning result report. Focusing on clinical cases, the corresponding tasks are completed through group discussion and collaboration, viewpoint exposition, role playing, situational simulation, etc. (2) Teachers organize teaching activities, put forward advanced tasks, guide and assist, comment, reflect and summarize in the process of students' activities, play a leading role, and focus on creating a good atmosphere for teamwork, and mobilize and stimulate students' enthusiasm and interest in learning, through peer-to-peer learning [31]. The role of discussion, inspiration and example between teachers and students, mutual influence and mutual promotion, improve students' clinical thinking and judgment ability, and complete knowledge internalization. (3) Evaluation, including group evaluation, self-evaluation, peer evaluation and teacher evaluation, so that students have a correct understanding of their entire learning process.

From Figure 3, it can be seen that under the clinical case teaching mode, teachers' teaching pays more attention to the cultivation of students' abilities, which enlarges the proportion of ability cultivation in the classroom.

(c) Afterschool extension

Teachers assign tests and homework based on students' learning in the first two stages, and issue expansion tasks to students who have spare capacity for learning. The main content is reflection and suggestions on the case [32] Although the core of the clinical case teaching method is to take the classroom as the main position for cultivating students' thinking ability, it also puts forward higher requirements for teachers' inspiring and guiding role. Some experiments in the research show that in the early stage of the implementation of the clinical case teaching method, the teacher's demonstration analysis of the case is very important. When they first came into contact with clinical cases, most students were very nervous and excited, and few students could actively analyze and verify the cases based on their theoretical knowledge. At this time, teachers are required to guide students to analyze from multiple angles according to the characteristics of the demonstration cases and find out whether they can summarize more scientific nursing countermeasures through group discussion [33].

As can be seen from Figure 4, the teaching activities of teachers after class can be mainly divided into three parts: layout test, postexpansion tasks, and monitor learning. Compared with the past, teachers' afterschool teaching activities are more targeted and more efficient.

#### 2.2.2. Teaching Method of the Control Group

In a preselected control group, teachers employed traditional teaching formats. The specific process is to divide the students into 8 groups with 6 students in each group (5 students in the eighth group). The day before the class starts, the teacher asks the students to preview the relevant knowledge, first teaches the theoretical knowledge during the class, displays the relevant practice of the theoretical knowledge through PPT, etc., and emphasizes the details that need to be paid attention to in the knowledge points. Finally, afterclass thinking questions are assigned to students.

### 2.3. Teaching Evaluation

Evaluation methods include course performance evaluation and questionnaire feedback analysis.

The performance evaluation of gynecological nursing course consists of process evaluation (50%) and summative evaluation (50%). Among them, the process evaluation includes classroom participation (10%, including group evaluation, self-evaluation, peer evaluation, and teacher evaluation), gynecological nursing skills operation assessment (20%), and stage theory test scores (20%). Summative assessment is the final theory test score, as shown in Table 1.

The questionnaire feedback analysis refers to the case teaching method classroom teaching quality evaluation scale compiled by Li et al. A total of 93 questionnaires were distributed, and the recovery rate was 100%.

### 2.4. Statistical Methods

SPSS 20.0 statistical software was used for statistical analysis of the data. The independent sample *t*-test was used for the results of the two groups of students' course results, and the *χ*^2^ test was used for the evaluation of the teaching effect of the two groups of students, and the test level was *α* = 0.05.

### 2.5. Classroom Teaching Effect Evaluation Results

As can be seen from Table 2, whether it is the classroom teaching effect evaluation results, and the scores obtained by the experimental group are higher than those obtained by the control group.

From the data in Table 3, it can be seen that the students in the experimental group generally showed a positive trend in their evaluation of the effect of classroom teaching. There are three dimensions of “contributing to the understanding and mastery of knowledge” and “conducive to the improvement of clinical thinking and judgment ability and analytical problem-solving ability.” In the remaining five dimensions, students' satisfaction level is above 90%, of which “facilitate mutual learning and discussion” with a 95.7% satisfaction rating, with a total of 44 students agreeing with this option.

In the control group, only 13 people agreed with the dimension “conducive to students' mutual learning and discussion,” accounting for 27.7%, and the variance with the experimental group reached 45.470. Between the experimental group and the control group, the smallest gap was [22, 23]. The dimension is “conducive to the understanding and mastery of knowledge,” and the variance is only 4.171.

## 3. Discussion

### 3.1. Analysis of the Performance of the Gynecological Nursing Courses of the Two Groups of Students

The results in Table 1 show that when the clinical case teaching mode is applied in gynecological nursing teaching, the students' process evaluation is significantly higher than the control group's process evaluation (91.80 > 88.74, *P* < 0.05), and the skill operation assessment score of the experimental group is significantly higher than that of the control group (91.85 > 86.28, *P* < 0.05); classroom participation in the experimental group was significantly higher than that in the control group (88.37 > 85.70, *P* < 0.05). It shows that in gynecological nursing teaching, especially in gynecological practical training teaching, the use of clinical cases is closely related to the clinical nursing tasks of obstetrics and gynecology [34, 35] and improves students' interest in learning and curiosity. At the same time, focusing on clinical cases, the task plan is completed in the form of teamwork, inquiry, and discussion, and the results are reported and shared in groups. Students' learning activities are embodied in two aspects: individual independent learning and team cooperation learning. The two complement each other, which can promote students to learn from each other, learn from, supervise and share, and give full play to their respective strengths. At the same time, teachers control the teaching process and difficulty, timely feedback students' learning results, and create opportunities for students to succeed, encourage students to build self-confidence, and improve students' classroom participation.

In addition, in the process evaluation of the experimental group, there was no significant difference between the theoretical test scores and the control group (*P* > 0.05), while the summative evaluation (final theoretical test) of the experimental group was significantly higher than that of the control group (83.17 > 78.55, *P* < 0.05). The reason should be related to the distribution of the question types of the two theoretical examination papers. The questions in the stage theory test are all multiple-choice questions, mainly A1-type questions, that is, each test question consists of 1 stem and 5 alternative answers. The stem appears as a single sentence in narrative form, and only 1 of the alternative answers is the best choice. The final theory test has a variety of questions, including medical record analysis, short answer questions, and other questions. At the same time, in addition to A1-type questions, the multiple choice questions also include A2-type questions (the best multiple choice questions of the case summary type, and the test question structure is composed of 1 Brief medical record as the question stem and 5 alternative answers to choose from, A3-type questions (the best multiple-choice questions for case groups, the structure of the questions is to begin to describe a patient-centered clinical situation, and then propose 2 to 3 related questions, each related to the initial clinical scenario, but with different test points and independent of each other). Therefore, the stage theory test mainly examines the students' mastery of theoretical knowledge, while the final theory test focuses more on the students' ability to complete the job tasks in clinical situations, combining theory with practice, making judgments through clinical thinking, using knowledge comprehensively and flexibly. The advantages of clinical case teaching mode applied to gynecological nursing teaching are reflected.

### 3.2. Analysis of the Results of Classroom Teaching Effect Evaluation

The results in Table 2 show that the students in the experimental group are more interested in learning whether they can stimulate their interest in learning, improve their self-learning ability, help in understanding and mastering knowledge, help in mutual learning and discussion, and help in the application of clinical nursing skills, and whether it is beneficial for communication and communication skills [36, 37]. The evaluation of the improvement of cooperation ability, the improvement of clinical thinking and judgment ability and the ability to analyze and solve problems, and the connection between theoretical knowledge and practical skills were significantly higher than those of the control group (*P* < 0.05), indicating the application of the clinical case teaching model. It can guide students to participate in activities such as analysis, cooperation, discussion, thinking, and expression, improve classroom teaching effects, exercise students' comprehensive ability, and better complete the tasks of gynecological nursing positions.

### 3.3. The Improvement of Students' Satisfaction with the Classroom

In gynecological nursing teaching under the traditional teaching mode, the learning of theoretical knowledge is too monotonous for students, and their subjective initiative in the learning process is very limited. The gynecological nursing major requires students' practical ability far higher than the theoretical basis, so most students are not satisfied with the traditional classroom. The selection of clinical case teaching not only fits the theme of classroom teaching but also represents typical cases. The theoretical basis and practical effects of the case are analyzed by the students themselves, the students' passive participation is transformed into active learning, the teacher's main responsibility is transformed from knowledge imparting to thinking and guidance, and the main way for students to improve is from mechanical memory to observation and understanding. The clinical case teaching model has changed the inherent way of teachers imparting knowledge to students in one direction, so that students can change from “I want to learn” to “I want to learn” in real situations, develop their thinking ability, and enhance their innovative awareness. To improve students' practical skills and theoretical knowledge application ability, stimulate students' interest in learning, improve self-study ability, exercise students' clinical thinking, analysis and problem-solving, teamwork and communication skills, and play an active role in gynecological nursing teaching, it is well received by students and is worthy of promotion.

## 4. Summary

Experiments have confirmed that the application of clinical case teaching in gynecological nursing teaching enables students to achieve significant growth from the mastery of theoretical knowledge to comprehensive practical skills. The survey of students and teachers shows that 77.8% of students and 83.4% of teachers hope to replace the traditional teaching mode with clinical case teaching and realize daily application in teaching. 82.3% of the students believed that the clinical case teaching method effectively enhanced their interest in professional learning and also promoted their mastery of theoretical knowledge and the combination of practical skills. This positive response from the students shows that the clinical case model can be universally applied to the daily teaching of gynecological nursing. But in practice, some problems are also exposed. For example, in the process of using clinical case teaching, the degree of “decentralization” of teachers should be limited, and whether too many cited cases to guide students to analyze will lead to inertia of teachers and students. For some students with weak self-control, how to ensure that they can play an applied role in the group, the above problems need to be explored and solved during the implementation of the clinical case teaching method. In the next step of research, the team will analyze the solutions to the above problems through the use of multiple clinical case teaching, hoping to provide more useful reference for the development of clinical case teaching in gynecological nursing teaching.

## Figures and Tables

**Figure 1:** Research process framework.

**Figure 2:** Teacher activities before class.

**Figure 3:** Teacher activities of classroom implementation.

**Figure 4:** Teacher activities of classroom implementation.

**Table 1:** Course grade evaluation.

Course grade evaluation	
Process evaluation	Summative evaluation
Class participation (10%); gynecological nursing skills operation assessment (20%); stage theory test score (20%)	Final theory exam

**Table 2:** Classroom teaching effect evaluation results.

Group	Summative evaluation	Process evaluation	Process evaluation subitems		
			Skill operation test	Class participation	Stage theory test
Test group (*n* = 46)	83.17 ± 5.092	91.80 ± 3.311	91.85 ± 5.842	88.37 ± 4.855	93.46 ± 7.865
Control group (*n* = 47)	78.55 ± 5.094	88.74 ± 4.062	86.28 ± 6.772	85.70 ± 4.086	92.72 ± 7.773
*t*	4.375	3.977	4.244	2.869	0.452
*P* value	<0.05	<0.05	<0.05	<0.05	>0.05

**Table 3:** The evaluation results of students in the experimental group and the control group on the teaching effect (number of people (percentage, %)).

Project	Experimental group (*n* = 46)	Control group (*n* = 47)	*χ* ^2^	*P*
1 Help to stimulate interest in learning	43 (93.5)	32 (68.1)	9.604	<0.05
2 Helps to improve self-learning ability	42 (91.3)	23 (48.9)	19.831	<0.05
3 Contribute to the understanding and mastery of knowledge	38 (82.6)	30 (63.8)	4.171	<0.05
4 Facilitate mutual learning and discussion	44 (95.7)	13 (27.7)	45.470	<0.05
5 Useful application of clinical nursing skills	41 (89.1)	29 (61.7)	10.048	<0.05
6 Conducive to the improvement of communication skills and cooperation skills	43 (93.5)	21 (44.7)	26.120	<0.05
7 Conducive to clinical thinking and judgment ability and analytical problem solving improvement of questioning ability	38 (82.6)	20 (42.6)	16.835	<0.05
8 Favorable linkages between theoretical knowledge and practical skills	42 (91.3)	32 (68.1)	7.710	<0.05

## Data Availability

The data used to support the findings of this study are available from the corresponding author upon request.
